The article "Effect of Pulse Indicator Continuous Cardiac Output Monitoring on Septic Shock Patients: A Meta-Analysis" was published in 2022. Journal: Comput Math Methods Med.

# Effect of Pulse Indicator Continuous Cardiac Output Monitoring on Septic Shock Patients: A Meta-Analysis

**DOI:** 10.1155/2022/8604322

**Published:** 2022-04-16

**Authors:** Bin Wang, Lijuan Cai, Bin Lin, Qiongxiao He, Xuejun Ding

**Affiliations:** Emergency Department, The Third Affiliated Hospital of Zhejiang Chinese Medical University, Hangzhou City, 310000 Zhejiang Province, China

## Abstract

**Background:**

Septic shock (SS) is the most common severe syndrome in the Intensive Care Unit (ICU). Enhancing the monitoring of hemodynamic indexes in SS patients carries huge clinical implications for reducing patient mortality. Recently, pulse indicator continuous cardiac output (PICCO) has been widely used in clinical practice, but its advantages than central venous pressure (CVP) in guiding the treatment of SS patients remains to be refined. Therefore, this study is aimed at assessing the clinical effects of PICCO in the treatment of patients with SS.

**Methods:**

The authors systematically searched several databases (PubMed, EMBASE, Cochrane Library, and China National Knowledge) between January 2001 and February 2021. When searching for relevant articles, the authors combined the following phrases describing the monitoring group (“pulse indicator continuous cardiac output,” “central venous pressure”) with the disease of interest as well as management (“SS,” “sepsis”). The outcomes were independently assessed by two reviewers who scored the articles for methodological quality using the Cochrane Collaboration's “risk of bias” tool. Forest plots, as well as sensitivity and bias analyses, were carried out for the included articles. The primary outcome measures were length of ICU stay, duration of mechanical ventilation, 28-day mortality, and fluid resuscitation volume.

**Results:**

Ten studies comprising 350 cases monitored with PICCO and 373 cases monitored with traditional CVP were eventually identified. PICCO-monitored patients were observed to be significantly associated with shorter ICU stay than CVP-monitored patients (MD: −3.04, 95% CI: −4.74 to −1.34, *P* = 0.0005), shorter time of mechanical ventilation (MD: −1.84, 95% CI: −2.80 to −0.87, *P* = 0.0002), and lower 28-day mortality (RR: 0.67, 95% CI: 0.48 to 0.94, *P* = 0.02). The two groups showed no significant difference in subgroup analysis for fluid resuscitation volumes (*P* > 0.05).

**Conclusion:**

PICCO monitoring technique can significantly improve the prognosis of SS patients, shorten the time of mechanical ventilation and ICU stay, and reduce the 28-day mortality, which has positive guiding significance for patients with SS. Given the limitations of the quantity and quality of included studies, further research is warranted to verify the conclusions.

## 1. Introduction

Septic shock (SS) refers to the manifestations of shock caused by various pathogenic bacteria and their toxins, most of which are clinically severe [1]. Pathogenic bacteria or their secreted toxins invade the blood circulation, which results in the production of various cytokines or mediators in the body, causing metabolic disorders, dysfunction, and SS [2, 3]. The common pathogenic bacteria causing SS are Escherichia coli and Klebsiella found in Gram-negative bacteria, as well as hemolytic streptococcus and Staphylococcus aureus found in Gram-positive cocci. Elderly people with diabetes, liver cirrhosis, cardiovascular and cerebrovascular diseases, and immune system diseases are more susceptible to SS. Infants are also at high risk for SS [4–6].

SS, the most common severe syndrome in the Intensive Care Unit (ICU), can lead to hemodynamic instability and impaired cardiovascular function in patients [7, 8]. In severe cases, patients often develop refractory hypotension and cardiovascular failure, eventually leading to death. Patients with SS require sufficient fluid resuscitation to ensure fluid circulation, but excessive fluid load can lead to multiple organ edema and even death [9–11].

Enhancing the monitoring of hemodynamic indexes in patients with SS has great significance to reduce the mortality of patients [2, 12], which is also the reason and clinical implications of this study. Venous pressure, dynamic pressure, volume index, and even microcirculation perfusion can be used for resuscitation monitoring. Central venous pressure (CVP) has been a common index for monitoring fluid resuscitation due to its simplicity of measurement; although, it cannot accurately reflect cardiac preload [12, 13]. Pulse indicator continuous cardiac output (PICCO) monitoring, on the other hand, is a novel technique that has emerged in recent years and has been recognized by ICU doctors due to its involvement of more indicators and high accuracy [14–16].

PICCO monitoring is a new technique combining pulse contour continuous cardiac output and pulmonary thermodilution cardiac output. Research has shown that the monitoring indicators can better reflect the volume state of patients [17–19]. PICCO has been widely used in clinical practice in recent years. Invasive monitoring of hemodynamic parameters to guide fluid therapy in SS patients is the research focus in this field [20, 21]. However, it is not clear whether PICCO is superior to CVP in guiding SS treatment [22, 23].

Accordingly, a meta-analysis was carried out to clarify the effect of PICCO in the treatment of SS patients, aiming at providing a theoretical basis for its clinical application.

## 2. Data and Methods

### 2.1. Literature Retrieval Strategy

We systematically searched PubMed, EMBASE, Cochrane Library, and China National Knowledge databases from January 2001 to February 2021 using the following keywords: (1) pulse indicator continuous cardiac output (PICCO), (2) central venous pressure (CVP), and (3) septic shock (SS), all of which were combined with the Boolean operator “and.” In the literature search, we set no restrictions on the language of publication. The reference list of the retrieved articles was also manually filtered to further identify potentially relevant studies that might have been missed by the retrieval strategy.

### 2.2. Study Selection

Studies were selected based on the following inclusion criteria:

1. Patients with SS
2. Patients monitored by PICCO were assigned to the experimental group (PICCO group), and those monitored by traditional CVP were set as the control group
3. Containing indicators assessing efficacy of the PICCO group and CVP group (control group)
4. Full-text articles were available
5. Prospective clinical studies, retrospective observational studies, or randomized controlled trials (RCTs)

The exclusion criteria were as follows:

1. Research on other diseases
2. Patients with other monitoring technology
3. No relevant data reported
4. Articles that are incomplete or full text unavailable

### 2.3. Data Acquisition and Quality Assessment

For potentially eligible studies, two reviewers independently check the eligibility of full-text articles using standard forms after title and abstract screening and extracted the following data from each eligible study: the first author's name, research type, patient age and gender, year of publication, sample size, study duration, and primary outcomes (length of ICU stay, duration of mechanical ventilation, 28-day mortality, and fluid resuscitation volume). Any conflicts were resolved by consensus or by a third reviewer. The Cochrane Collaboration's “risk of bias” tool was used for methodological quality assessment of the included studies [24].

### 2.4. Statistical Analysis

Meta-analysis was carried out with the use of Review Manager (*v*5.3, Cochrane Collaboration, 2014). The results were presented as forest plots, and *P* < 0.05 was defined as statistical significance. Mean difference (MD) and 95% confidence interval (CI) were calculated for continuous data, with risk ratio (RR) and 95% CI for binary data. Statistical heterogeneity among the included studies was tested using the *χ*^2^, *I*^2^, and Tau^2^ statistic. Significant heterogeneity was rendered as *P* < 0.05 or *I*^2^ > 50%. And the formula for *I*^2^ was *I*^2^ = (*Q* − df)/*Q* · 100%, where *Q* is *χ*^2^ and df is the degree of freedom. *I*^2^ values of 25%, 50%, and 75% are considered low, moderate, and high estimates, respectively. Results were analyzed using a fixed-effect model when heterogeneity was at a low estimates, while using random-effect model when heterogeneity was at a high estimates. Funnel plots were used to assess publication bias based on standard errors (SE) and corresponding measures. A *P* value ≤0.05 was considered statistically significant.

## 3. Results

### 3.1. Search Process

A total of 714 studies were identified through the retrieval strategy. A careful screening revealed 85 eligible studies, of which 75 were further excluded because of different research design or data insufficiency. Eventually, 10 complete papers meeting the selection criteria were included in this meta-analysis [25–34].  Figure 1 illustrates the search process with eligibility criteria.

### 3.2. Characteristics of Included Studies

The 10 eligible articles, which included 7 RCTs, 2 prospective clinical studies, and 1 retrospective observational study, were published between 2014 and 2020. A total of 723 patients were included in the meta-analysis, including 350 cases monitored by PICCO and 373 by traditional CVP. The primary outcome measures were length of ICU stay, duration of mechanical ventilation, 28-day mortality, and fluid resuscitation volume (Table 1).

### 3.3. Quality Assessment

The methodological quality of the 10 articles was evaluated using the Cochrane's risk of bias tool. Two out of the 10 included studies were reported of high risk of performance bias and reporting bias (Figure 2). See Figure 3 for the risk of bias assessment for each study.

### 3.4. Results of Heterogeneity Test

Eight studies comprising 282 patients in the PICCO group and 305 patients in the control group reported the length of ICU stay. The forest plot showed significantly reduced ICU stay in the PICCO group compared with the control group using the random-effects model (MD: -3.04, 95% CI: [-4.74, -1.34], *P* = 0.0005), indicating significant heterogeneity (*P* < 0.00001, *I*^2^ = 92%) (Figure 4). This conclusion was still valid after sensitivity analysis excluding Xu's 2014 study (*P* < 0.00001, *I*^2^ = 69%).

The duration of mechanical ventilation was reported in 613 patients in these 8 studies. Meta-analysis revealed that the mechanical ventilation time in PICCO-monitored patients was shorter than that in CVP-monitored patients (MD: -1.84, 95% CI [-2.80, -0.87], *P* = 0.0002, random-effects model), with significant homogeneity among the included studies (*P* < 0.00001, *I*^2^ = 81%) (Figure 5). This conclusion was still valid after sensitivity analysis excluding Huang's 2017 study (*P* = 0.0002, *I*^2^ = 55%).

Regarding the 28-day mortality, 7 studies (249 in the PICCO group and 254 in the control group) provided relevant information. The heterogeneity of 28-day mortality assessed by the fixed-effect model identified a significant difference in 28-day mortality between the PICCO group and CVP group (RR = 0.67 with 95% CI [0.48, 0.94], *P* = 0.02), while no significant heterogeneity among the included studies (*P* = 0.46, *I*^2^ = 0%) (Figure 6).

A subgroup analysis was performed to evaluate the heterogeneity of fluid resuscitation volumes at different time points, taking into account changes in fluid resuscitation over time. The 8 trials were first divided into three subgroups (6 h, 24 h, and 48 h). It was found that there was no significant difference between groups in subgroup analysis for fluid resuscitation volumes (*P* > 0.05); although, significant heterogeneity was present in included studies. Sensitivity analysis also showed robust results (Table 2).

### 3.5. Publication Bias

The publication bias was assessed based on the 28-day mortality. It was found that the funnel plot of 28-day mortality was symmetrical, suggesting the absence of significant publication bias in this meta-analysis (Figure 7).

## 4. Discussion

Sepsis is a life-threatening organ dysfunction attributed to the dysregulation of the body's response to infection, according to the latest sepsis guidelines in 2016. Evidence has shown that SS is responsible for 25%-70% of in-hospital mortality [13, 35, 36]. Early fluid resuscitation within 6 hours after the episode is the key to SS management. Coen's study confirmed that early active fluid resuscitation treatment can significantly reduce the mortality of patients [37]. To prevent SS, attention should first be paid to the treatment of etiology, that is, to actively fight infection, such as the use of sensitive antibiotics [38, 39], which could improve the function of vital organs and maintain the balance of blood vessels [40].

The early goal-directed therapy (EGDT) proposed by Rivers emphasized rapid volume expansion to increase cardiac output and oxygen supply, which can rapidly restore circulating blood volume, and shorten the duration of hypoperfusion in tissues and organs [41, 42]. The EGDT protocol aims to achieve resuscitation within 6 hours after the onset of SS, which contributes to significantly reduced mortality and incidence of multiple organ dysfunction [18, 43].

According to the EGDT protocol, patients with SS need to reach a CVP of ≥1.07-1.60 kPa within 6 hours. However, CVP is easily affected by many factors such as cardiovascular compliance, intrapleural pressure, and mechanical ventilation, which cannot accurately reflect the state of cardiac preload. In order to maintain the relative stability of circulation in patients with SS, early targeted volume resuscitation should be advocated [18, 44].

Early identification, timely diagnosis, and effective prevention and treatment, as well as optimization of treatment strategy are the key to improving the success rate of SS treatment [45, 46]. PICCO monitoring technology, a clinical method for monitoring hemodynamics, can comprehensively reflect the changes of hemodynamic parameters and cardiac systolic and diastolic function, which has guiding significance for volume resuscitation, fluid management, diuretic application, and efficacy judgment in patients with shock [47–49].

PICCO combines pulmonary thermodilution with arterial pulse waveform analysis technology, which can dynamically monitor functional hemodynamic parameters and effectively evaluate the volume status of patients [50, 51]. It has now become an important blood flow monitoring method in the treatment of SS and can guide fluid resuscitation and accurately determine volume responsiveness [52–54]. Studies have shown that PICCO technology can guide volume management and the use of vasoactive drugs by evaluating cardiac preload and can avoid volume overload and pulmonary edema during treatment while ensuring normal tissue and organ perfusion [55–57].

The study of Schneck et al. showed that for SS patients with myocardial injury, PICCO-guided fluid resuscitation can reduce the occurrence of fluid overload, reduce the degree of organ dysfunction, and shorten the duration of mechanical ventilation and ICU stay [58]. CVP is used as an indicator to evaluate the state of vascular volume because of its simplicity, but some studies have shown that CVP is not significantly correlated with blood volume [59, 60]. Xie et al. reported that severe SS often led to myocardial depression, and early recognition, early monitoring, early judgment of cardiac insufficiency in SS, and timely correction can improve the prognosis of patients [17, 44, 61]. Some patients cannot tolerate high-dose fluid resuscitation in a short time due to the effect of SS on cardiac function, while PICCO can simultaneously monitor cardiac function indexes such as dPmax, SVI, and cardiac output index (CI); once patients have poor cardiac function, dobutamine can be timely used for cardiotonic therapy to improve their cardiac function, allowing patients to tolerate more fluid load in a short time [59, 62, 63].

Ten studies involving 723 patients with SS were enrolled. The results showed that the duration of mechanical ventilation and ICU stay in the PICCO group was significantly shorter than that in the control group (*P* < 0.05), which was consistent with the study of Ameloot et al. [55]. It also indicates that, compared with traditional CVP treatment, PICCO can reduce the disease severity of SS patients, more accurately guide fluid resuscitation, reduce lung water, and shorten the duration of mechanical ventilation and ICU stay. In addition, a significant difference was observed in the 28-day mortality between the two groups (*P* < 0.05), which was similar to the results of three large randomized trials [52, 64, 65]. Therefore, PICCO monitoring technology has more advantages than traditional CVP monitoring technology and can significantly improve the prognosis of patients. However, there are currently few international studies on PICCO monitoring technology to guide SS; so, the application value of PICCO in ICU hospitalized SS patients needs further study.

This study still has some limitations. First, the sample size of nine of the ten studies we analyzed was small (less than 100), and there may be some errors in the test results. Second, there are some unpublished and missing data in the studies included in the analysis, which may lead to a bias against the pooled effect. We will address these limitations in future research.

## 5. Conclusion

This meta-analysis shows that PICCO monitoring has a positive impact on the prognosis of SS patients, which can effectively shorten the duration of mechanical ventilation and ICU stay, accurately guide fluid resuscitation, and significantly improve the 28-day survival of patients, providing new insights into the monitoring and management of SS patients.

## Figures and Tables

**Figure 1:** Flow chart of study selection.

**Figure 2:** Risk of bias of included studies: low (green), unclear (yellow), and high (red).

**Figure 3:** Summary of risk of bias.

**Figure 4:** Forest plot: comparison of length of ICU stay.

**Figure 5:** Forest plot: comparison of duration of mechanical ventilation.

**Figure 6:** Forest plot: comparison of 28-day mortality.

**Figure 7:** Forest plot: comparison of hospital length of stay.

**Table 1:** Characteristics of included studies.

Study	Study design	Gender (M/F)		No. patients		Age		Years of onset	Primary outcome^∗^
		PICCO	Control	PICCO	Control	PICCO	Control		
Liu et al. 2017	RCT	20/10	19/11	30	30	56 ± 9.5	54 ± 10.1	September 2015 to July 2017	1, 2, 3, 4
Lu et al. 2015	Prospective clinical study	35/17	33/19	53	52	60.8 ± 15.1	61.5 ± 14.4	Unclear	1, 2, 3, 4
Wang et al. 2020	Prospective clinical study	23/20	33/18	43	51	65.9 ± 10.4	64.6 ± 11.7	March 2017 to February 2020	1, 2, 3, 4
Ma et al. 2017	RCT	15/5	14/6	20	20	77.9 ± 6.5	76.6 ± 6.7	January 2013 to December 2015	1, 2, 3, 4
Liu et al. 2016	RCT	14/11	15/10	25	25	46.3 ± 7.9	45.7 ± 8.9	August 2012 and August 2013	4
Xu et al. 2014	RCT	18/12	16/12	30	28	49 ± 13	47 ± 11	March 2011 to March 2013	1, 2, 3, 4
Li et al. 2020	Retrospective observational study	/	/	30	30	34.0 ± 8.7	35.1 ± 8.6	July 2014 to July 2020	1, 3
Mutalipu et al. 2014	RCT	21/11	32/18	32	50	50.5 ± 12.3	54.9 ± 14.6	January 2013 to July 2014	1, 2, 4
Yao et al. 2017	RCT	23/21	24/20	44	44	63.5 ± 8.5	62.6 ± 7.4	February 2016 to May 2017	1, 2
Huang et al. 2017	RCT	25/18	26/17	43	43	63.5 ± 8.2	63.9 ± 9.0	January 2011 to December 2015	2, 3, 4

^∗^1: length of ICU stay; 2: duration of mechanical ventilation; 3: 28-day mortality; 4: fluid resuscitation volume. RCT: randomized controlled trial.

**Table 2:** Forest plots result: comparison of fluid resuscitation volumes.

Subgroup analysis	*N*	MD(95% CI)	*P* values	Test for heterogeneity		
				Chi^2^	*P*_*h*_	*I* ^2^
Fluid resuscitation volumes (mL)						
6 h	8	178.50 (-255.82, 612.82)	0.42	240.36	<0.00001	97%
24 h	8	-197.27 (-1334.32, 939.79)	0.73	642.02	<0.00001	99%
48 h	4	-693.25 (-1434.88, 48.38)	0.07	19.22	0.0002	84%

N: number of trials; MD: mean difference; CI: confidence interval; Ph: *P* value of the *Q* test for heterogeneity.

## Data Availability

The labeled dataset used to support the findings of this study are available from the corresponding author upon request.
